# A Descriptive Case Study of Skilled Football Goalkeepers During 1 v 1 Dyads: A Case for Adaptive Variability in the Quiet Eye

**DOI:** 10.3389/fpsyg.2022.908123

**Published:** 2022-07-07

**Authors:** Benjamin Franks, William M. Roberts, John Jakeman, Jonathan Swain, Keith Davids

**Affiliations:** ^1^Sport, Exercise and Physical Activity Research Group (SEPARG), Faculty of Health and Life Sciences, Oxford Brookes University, Oxford, United Kingdom; ^2^Sport Exercise and Rehabilitation Sciences, Canterbury Christ Church University, Canterbury, United Kingdom; ^3^Te Huataki Waiora—School of Health, University of Waikato, Hamilton, New Zealand; ^4^Sport and Human Performance Research Group, Sheffield Hallam University, Sheffield, United Kingdom

**Keywords:** quiet-eye, perception—action, ecological dynamics, goalkeeping, football

## Abstract

Evidence investigating skilled performers in sport suggests that a prominent component of skilled behavior is, in part, due to the development of more effective and efficient perception-action couplings. Further, the Quiet Eye has emerged as a useful tool in which to investigate how skilled performers regulate action through fixating on visual information within the immediate environment before the onset of a goal directed movement. However, only a few contributions to the literature have attempted to examine the individual variations within these Quiet Eye fixations in skilled participants. In this case study, we first asked how goalkeepers control their actions, via the Quiet Eye in a representative task. Second, we sought to examine whether inter- and intra- individual differences in the Quiet Eye are present in skilled goalkeepers as a functional component of skilled performance. Results were consistent with previous work on football goalkeepers, with QE fixations located at the ball and visual pivot. However, individual analysis reveals different Quiet Eye gaze patterning between (inter) and within (intra) the goalkeepers during saving actions. To conclude, we have provided a descriptive case study in attempt to understand the Quiet Eye behaviors of a skilled sample of professional goalkeepers. In doing so we have suggested how adaptive variability, founded upon an Ecological Dynamics framework, may provide further insight into the function of the Quiet Eye.

## Introduction

A prominent component of skilled behavior is, in part, due to the development of more effective and efficient perception-action couplings. In comparison to less skilled individuals, highly skilled performers can identify key sources of visual information and use them to regulate actions, reciprocally using actions to generate new information (van der Kamp and Renshaw, 2015). An important aspect of skilled perception is using visual exploratory behaviors such as eye movements and fixations to discover, explore and exploit visual information to guide behavior (Williams et al., 1999, 2004).

Consequently, evidence suggests that successful performance can be determined by the specific visual search strategy deployed by a performer (for examples see Abernethy and Russell, 1987; Kato and Fukuda, 2002). Notably, the Quiet Eye (QE) has emerged as a particular perception-action variable that has illustrated this point. The QE is concerned with the final visual fixation, lasting over 100 ms at a single location, prior to the critical phase of a goal-directed movement (Vickers, 2007).

Coined by Vickers (1996), the significance of the QE is founded upon its ability to provide an insight into a specific information variable which couples perception and action. Consequently, the QE has been referred to as a core perception-action variable utilized across the sport, medical and development domains, and is considered an integral part of successful performance (Sun et al., 2016).

A particular case for the need to hold superior perception-action couplings is of goalkeepers within football. Primarily, goalkeepers are tasked with preventing the ball from entering the goal whilst under extreme temporal and spatial constraints (Piras and Vickers, 2011). In work conducted by Piras and Vickers (2011), goalkeepers attended to the visual pivot during the final stage of the strikers kicking action during penalty kicks. Further still, the authors found that if the QE fixation exceeded 1,100 ms, then the chance of a goal being scored increased.

The authors of the present paper have investigated the QE in football goalkeeping previously. In this work it was found how QE patterning is modulated by specific task constraints and their manipulation by experimenters (Franks et al., 2019). In our investigation, differences emerged between performance in the traditional football penalty kick (A static ball struck from a central position to the goal 11 m away) and performance in a representative dyadic task between a goalkeeper and shooter that is replicated in this paper. Specifically, differences were observed in the QE duration and the timing of the QE, with the relative onset occurring later in the representative task (21.13 ± 4.21% v 36.38 ± 4.30%) and subsequently offsetting later (73.48 ± 1.58% v 82.40 ± 3.79%).

Despite a general acceptance that variations in task constraints applied to experimental conditions may cause significant perceptual-motor adaptations in participants (Williams et al., 2004; Vaeyens et al., 2007; Dicks et al., 2010a; Rienhoff et al., 2016), one criticism proffered against research analyzing perception-action couplings, and in particular the QE, is the over-reliance on generalizations of mean group data (Renshaw et al., 2019). Group-based generalizations in this case, have led to an assumption of the existence of a putative “optimal perceptual strategy” (Caballero et al., 2019). However, analysis of individual differences in performance is considered important from the perspective of skill adaptation, reflecting how each individual explores and exploits variability in perception and action to self-regulate in performance environments (Araújo and Davids, 2011; Button et al., 2020).

Indeed, *adaptive variability* has been observed between individuals when studying visual search strategies during performance of dynamic interceptive tasks. Dicks et al. (2010b) demonstrated how specific action capabilities (effectivities) of a goalkeeper can result in different actions emerging within-individuals to utilize affordances (opportunities) to regulate interceptive actions. Results suggested that the relative differences in action capabilities (in this instance, response times) of a goalkeeper may support the utilization of a different perception-action coupling relationship, with quicker goalkeepers being able to pick up and use more action-specifying information closer to foot-ball contact to reduce error, whereas slower goalkeepers were recorded as needing to use information that emerged much sooner to regulate actions.

As well as the identification of *between-individual* variability in the use of visual search behaviors, variability *within-individuals* has also been observed. For example, Chia et al. (2017) explored variability of the QE duration in 10-pin bowling. They noted significant variance in the QE values, alluding to the functionality of the QE being dependent on the task-individual relationship and variability from the mean being indicative of adapting to task constraints (for original arguments; see Williams et al., 2004).

Previous research findings raise important questions on the role of inter- and intra- individual variability in QE strategies during skilled action. As such, in this descriptive case study we set out to provide a single subject (Bates, 1996) inter- and intra- individual analysis of QE behaviors in a sample of skilled football goalkeepers. We sought to adopt a case study approach, rather than a cross sectional design, because it allowed us to look more closely at a niche performance group allowing us to identify how highly skilled goalkeepers perform *in situ*. Likewise, using a single subject design allows us to capture the inherent variability existent in biological systems, offering a behavioral analysis that demonstrates each actor’s unique signature behavior under competing constraints (Newell and Corcos, 1993; Bates, 1996).

Indeed, because differential response patterns emerge through an individual’s different experiences and perceptions, an analytical approach must cater for such variations in behavioral solutions during the same task. Single subject research designs can cater for such variations in behavioral solutions during the same task (Bates, 1996). Often, qualitative changes in behavior escape the attention of traditional statistical analysis.

To summarize, whilst research investigating skilled coupling of perception and action increasingly represents *in situ* sporting situations, there are still methodological and philosophical concerns regarding the analysis of skilled behavior (Pinder et al., 2011a,b). Particularly, the averaging of QE data toward a putative optimal point for successful performance may not cater for individual performer differences and their effectivities (Gibson, 1979; i.e., capacities and capabilities). These results may have led to a limited interpretation of data falling to either side of the mean, which may be evidence of functionally adaptive variability and of a highly flexible and skilled coupling of perception and action. Here, we discuss evidence from a case study, drawing on a sample of highly skilled professional football goalkeepers, seeking to investigate the QE behaviors under representative task constraints during a 1v1 dyadic task, typically faced in competition and practice.

In doing so, we expected that inter- and intra- individual variability would be manifest in QE values, implying that a sample of skilled goalkeepers’ performance can be characterized through the formation of more flexible and skilled perception-action couplings in light of representative task constraints.

## Materials and Methods

### Participants

Participants (*n* = 4) were all adult male, skilled, professional football goalkeepers (26.3 ± 4.2 years) who were convenience sampled for the study. The parameters for categorizing participants as skilled included that, at the time of data collection, they were above the age of 18 years and employed as a goalkeeper for a full-time professional football club in the United Kingdom. The sampled players had a mean of 5.7 ± 3.1 years of full-time professional playing experience. All participants had normal or corrected to normal vision and gave their informed written consent to participate in the study after institutional ethical approval (DREC Reference 0417-42) was granted on the basis of adhering to the declaration of Helsinki guidelines for dealing with live participants.

### Apparatus

A head-mounted SensoMotoric eye movement registration system (SMI-ETG) (SensoMotoric Instruments, Inc., Boston MA) recorded the participants eye-movements. A SONY HDR-PJ410 Digital HD Video Recorder was mounted at 153 cm height to film the actions of the participants and the ball path. Goal areas at the respective football clubs training facility were used to ensure familiarity, and consistency with Football Association standards. Gaze data from the SMI-ETG were exported via the BeGaze software (Tracksys, Nottingham) at 60 Hz frame rate. For calibration, the manufacturer’s procedures for specification of a 1-point calibration was followed and repeated after every 5 actions, or when requested by the goalkeeper if the glasses had slipped. When evidence of the inordinate movement of the glasses (through slippage or a knock) emerged, the trial was discarded, and an additional trial was undertaken.

### Protocol

Three self-reported right-footed, male kickers (23 ± 2.7 years) from the same professional football clubs as the goalkeepers volunteered as participants to take part in the study as the shooters. The kickers had a mean of 3.1 ± 0.6 years of experience at the professional level. A shooter v goalkeeper *in situ* dyadic system (1v1) was created to replicate the demands of a typical goalkeeper performance environment.

A dyadic system interaction is common in team games and has been used previously when studying the actions of goalkeepers in football (e.g., Shafizadeh et al., 2016). The dyadic system is used here to describe the 1 v 1 relationship that the kicker and goalkeeper engage in during the task.

The goalkeeper, stood on the goal line in the center of the goal, would signal when ready to initiate the trial, inviting the shooter to travel with the ball from a fixed point 20 m from the goal line and having to strike the ball when they reached the shooting line at 11 m (Figure 1). The shooter was encouraged to score quickly to replicate a pressured scoring situation.

**FIGURE 1:** The experimental set up of the 1 v 1 dyadic task. **(A)** The goalkeeper; **(B)** shooting line at 11 m; **(C)** the start line at 20 m; **(D)** the Shooter; **(E)** external SONY HDR-PJ410 Digital HD Video Recorder; **(F)** football goal to FIFA requirements.

The recorded trials took place over 3 sessions during the course of a season with no more than 30 trials (including 10 familiarization trials) being recorded per session to avoid mentally and physically fatiguing participants. The trials were presented in blocks of 5, with each goalkeeper being provided a rest period of their own choosing and asked only to set for the next block once they felt comfortable and without any immediate effects of fatigue. The 3 sessions took place at the start of each clubs pre-season phase (Between week 1 and 2 of each clubs respective pre-season), the end of the pre-season phase (Between week 5 and 7 of each clubs respective pre-season) and the final session during the season between game week 11 and 16. Session 1 yielded 14.5 ± 1.91 recorded trials, session 2 11.25 ± 1.89 and session 3 4.25 ± 1.26.

### Dependent Variables and Analysis

Gaze behaviors and movement data were coded following procedures adopted from Klostermann et al. (2018), via a manually created Vision-In-Action system (VIA). The exported BeGaze eye tracking video file was time-synchronized with the external scene camera video file through a commercially available editing tool to create a split screen of the gaze and motor behaviors (Filmora, v7.8; WONDERSHARE, LHASA).

The movement phases (defined using Piras and Vickers, 2011) were identified for the goalkeeper as General Preparation (GPrep): onset of trial to onset of hop; Hop (Hop): offset of hop to ball contact; Reaction time (Rt): ball contact to first movement to save the ball; and Movement time (Mt): offset of RT to trial offset.

The start of the trial was categorized as the shooter’s first step in the direction of the ball. The end of the trial occurred when the ball was intercepted by the Goalkeeper, entered the goal, or left the pitch. The QE fixation was deemed to occur when the participant’s gaze was stabilized on a particular location within 3° of visual angle or less for a minimum of 100 ms. The QE period was deemed to have occurred at the start of the hop phase (Ghop) of the goalkeeper’s movement (Piras and Vickers, 2011).

Two fixation locations were identified, drawing on consistent findings in the literature and through observations of the participants’ gaze locations: the ball and the visual pivot (VP). The VP is defined in which the gaze “is centrally located between the ball and kicking leg, thus enabling the optimal use of both the foveal and parafoveal vision” (Piras and Vickers, 2011; p. 246).

The QE onset, offset and duration values were analyzed for shots saved and scored with a Wilcoxon Signed Rank test. QE mean onset, offset and duration were analyzed for shots saved and scored with a Wilcoxon Signed Rank test. QE onset, offset and duration values were analyzed across the two locations observed (ball and VP) with a Wilcoxon Signed Rank test. Individual Goalkeeper’s QE onset, offset and duration values were analyzed for fixation location with a Wilcoxon Signed Rank test.

Functional adaptive variability was characterized by the variability observed between individual goalkeepers (inter-individual variability) and within individual goalkeepers (intra-individual variability) in successful trials (tasks ending in a saving action). Functional adaptive variability for QE onset, offset and duration between individuals were analyzed using a Kruskal-Wallis *H*-test. Inter-individual variability for goalkeeper movement phases were analyzed using a Kruskal-Wallis *H*-test. Statistical significance levels are presented with adjusted *post hoc* Bonferroni correction. A simple linear regression was used to examine the relationship between QE gaze location by timing of the QE fixation, individually for both onset and offset. To observe functional adaptive variability within individual goalkeepers, a descriptive trial-by-trial analysis of individual QE profiles, using single subject scatter plots and standard deviations from the mean, is presented to show qualitatively different behaviors underpinning skilled performance with the sample of expert athletes.

## Results

Data were collected from a total of 120 trials, of which 13 trials were discarded due to technological faults, unclear eye tracking data or poor video quality. The mean length of trials totaled 1568.5 ms (± 158.38 ms). Due to a high standard deviation (± 10.1% of the total trial time) all results are presented as a relative time (%). Utilizing relative conversions has been used previously in QE research (Lebeau et al., 2016), for example Causer et al. (2010) used relative QE due to the variances in shot times. Analysis was conducted on trials ending in goals and saves (GK1 = 13, GK2 = 17, GK3 = 14, GK4 = 14) out of the total of 30 trials collected. In total, 58 of the 107 trials ended in saves (54.17%), with only small performance variations across all 4 goalkeepers (± 1.75%).

### Group Mean Analysis of Quiet Eye in Saves v Goals

Values for QE duration did not differ significantly between shots scored and shots saved by the participants (*p* = 0.223; saves = 45.65 ± 7.11%, goals = 49.15% ± 18.45%). However, values for QE onset differed significantly (*z* = –3.999, *p* = 0.000) with the QE onset occurring later in saves (36.38 ± 4.35%) than in trials resulting in a goal (24.00 ± 4.53%). QE offset occurred significantly later (*z* = –2.870, *p* = 0.004) during saves (82.40 ± 3.79%) than in goals (72.95 ± 7.13%).

### Individual Mean Analysis of Quiet Eye in Saves v Goals

There were no significant differences for QE duration between goals and saves for any of the participants (Table 1). However, the QE onset occurred significantly later in saves than in goals for goalkeeper 1 (*z* = –3.084, *p* = 0.003), 2 (*z* = –1.558, *p* = 0.041) and 3 (*z* = –2.039, *p* = 0.021), but not for goalkeeper 4 (*p* = 0.064). The offset of the QE revealed significant differences between saves and goals for goalkeeper 2 (*p* = 0.018) only, with a later offset in saves.

**TABLE 1:** Individual mean % Quiet Eye characteristic for Goals v Save and within individual Goal v Save Wilcoxon Signed Rank test.

	Duration			Onset			Offset		
Participant	Save	Goal	*P*=	Save	Goal	*P*=	Save	Goal	*P*=
GK1	44.47 ± 6.94	43.91 ± 6.70	0.657	34.26 ± 6.32	20.58 ± 9.55	0.003	78.73 ± 10.26	64.49 ± 15.82	0.075
GK2	46.72 ± 9.03	50.42 ± 20.83	0.778	32.74 ± 8.53	19.61 ± 16.58	0.041	79.66 ± 6.07	70.32 ± 17.24	0.018
GK3	45.68 ± 5.75	47.39 ± 15.74	0.534	40.79 ± 4.52	30.62 ± 17.66	0.021	86.48 ± 5.68	78.01 ± 17.12	0.091
GK4	45.39 ± 5.49	53.29 ± 17.62	0.133	39.35 ± 5.47	27.70 ± 16.96	0.064	84.74 ± 4.69	81.00 ± 10.03	0.221

### Inter-Individual Variability of Quiet Eye

Significant inter-individual variance was not demonstrated for QE duration (*p* = 0.912). However, significance was evident for the QE onset [X^2^(2) = 11.938, *p* = 0.008]. Goalkeeper 2 displayed the earliest mean QE onset, and Goalkeeper 3 showing the latest mean QE offset (Table 1). Significant differences were also observed for QE offset [X^2^(2) = 10.987, *p* = 0.012], with Goalkeeper 1 displaying the earliest mean QE offset, and Goalkeeper 3 the latest mean QE offset (Table 1).

### Inter-Individual Variability in the Location of the Quiet Eye Fixation

There were no significant differences between the duration of the QE fixation at the ball or the VP (*p* = 0.212). Analysis of the timing of the QE revealed that for the onset of the fixation (*z* = –4.076, *p* = 0.000) and the offset of the fixation (*z* = –4.349, *p* = 0.000), there were significant differences between fixations located on the ball or the VP. In both instances the QE fixation at the ball occurred later than the VP (Onset, 40.23 ± 3.67% v 32.76 ± 2.21; Offset, 87.13 ± 2.26% v 77.99 ± 5.38%). A simple linear regression was calculated to predict the QE gaze location based on the timing of the QE fixation, for either onset or offset. For location (visual pivot, or ball) by timing of onset, a significant regression equation was found [*F*(1, 56) = 29.905, *p* < 0.000], with an *R*^2^ of 0.348. As such, the model is able to demonstrate the goalkeepers gaze location is equal to 23.272 + 8.700 (onset) location being more likely to be placed on the ball when timing occurred later into the trial. By timing of offset, a significant regression equation was found [*F*(1, 56) = 46.111, *p* < 0.000], with an *R*^2^ of 0.452. The model is therefore able to demonstrate the goalkeepers gaze location is equal to 66.471 + 10.294 (offset) location being more likely to be placed on the ball when timing occurred later into the trial.

Variability was evident in the weighting of fixation locations by the goalkeepers. Goalkeeper 1 and 2 fixed their gaze at the VP more frequently than the ball (61.51 v 38.46% and 51.82 v 41,18%) and Goalkeeper 3 and 4 fixated the ball more frequently (71.43 v 28.57% and 64.29 v 35.71%).

### Inter-Individual Variability in Movement Phases

Within group analysis revealed significant differences between individuals for participant movement phases. Significant differences were demonstrated for GPrep [X^2^(2) = 24.574, *p* = 0.000]; GHop [X^2^(2) = 8.426, *p* = 0.038]; Rt [X^2^(2) = 45.887, *p* = 0.000], and Mt [X^2^(2) = 17.066, *p* = 0.001]. Goalkeepers 1 and 2 initiated movements earlier than Goalkeeper 3 and 4 (43.51 and 43.43% v 48.99 and 49.61%, respectively). Similarly, Goalkeepers 1 and 2 appeared to be slower movers, reporting longer Rt (14.36 and 15.11% v 12.49 and 14.09%) and longer Mt values (32.61 and 32.48% v 29.24 and 27.20%, respectively).

### Intra-Individual Variability in the Quiet Eye Effect

Intra-individual variability was demonstrated through the presentation of trial-by-trial analysis. Table 2 presents the mean QE values for duration, onset and offset. However, variability from the mean is illustrated in the relatively high standard deviations for each Goalkeeper (Figure 2).

**TABLE 2:** Individual mean % of movement phases for successful trials.

	GPrep	GHop	Rt	Mt
Mean	46.57 ± 2.81	8.90 ± 0.18	14.20 ± 1.06	30.33 ± 2.05
GK1	43.51 ± 3.40	9.52 ± 0.44	14.36 ± 0.36	32.61 ± 3.25
GK2	43.43 ± 3.20	8.98 ± 0.52	15.11 ± 0.41	32.48 ± 3.18
GK3	48.99 ± 2.83	9.28 ± 0.56	12.49 ± 0.56	29.24 ± 2.96
GK4	49.61 ± 4.69	9.10 ± 0.39	14.09 ± 0.51	27.20 ± 4.32

**FIGURE 2:** Inter-individual variation showing the relative (%) start time of the QE onset and corresponding offset of the QE fixation.

The mean QE duration for goalkeeper 1 for trials ending in a save totaled 44.47% with a standard deviation of 6.94%. However, as depicted from individual trials no single trial led to a QE duration of the same value. As illustrated in Figure 4, high levels of variability were present in saved trials varying from a duration of 26.84% in trial 1–53.97% in trial 12. This trend was also reflected for both QE onset (Mean onset 34.36%) where the standard deviation was again relatively high at 6.32% and QE offset (Mean offset 78.73%) with a standard deviation of 10.26%. There was also variability on the specific locations the QE fixation attended to. In trial 4, for example, the QE fixation attended to the ball onsetting 39.78% into the trial and offsetting at 87.86% of the trial. Yet, in trial 8 the QE onset at 28.26% and offset at 71.05% whilst the fixation attended to the visual pivot.

**FIGURE 3:** **(A)** A 95% confidence ellipse illustrating the timing (QE onset × QE offset) of the QE fixation at the VP. X denotes the group mean, • denotes each individual data point. **(B)** A 95% confidence ellipse illustrating the timing (QE onset × QE offset) of the QE fixation at the ball. X denotes the group mean, • denotes each individual data point.

**FIGURE 4:** Individual Goalkeeper Quiet Eye profiles demonstrating adaptive variability. **(A)** Goalkeeper 1 **(B)** goalkeeper 2 **(C)** goalkeeper 3 **(D)** goalkeeper 4. X denotes the group mean, • denotes each individual data point.

In contrast, goalkeeper 3 demonstrated lower levels of standard deviation, and therefore variability. The mean QE duration for goalkeeper 3 for saved trials was 45.68% with a standard deviation of 5.75%. For QE onset (mean onset 40.79%) lower levels of standard deviation emerged (± 4.52%) and similarly for QE offset (± 5.68%). Again, the location of the QE fixation did demonstrate flexibility in the QE strategy used. In trial 4 the goalkeeper onset the QE fixation at the visual pivot 47.43% into the trial and offset 91.60% in. Whilst in trial 7 the goalkeeper attended to the ball 33.84% into the trial and offset their gaze 75.47% in.

## Discussion

### Variability Within the Quiet Eye Expertise Effect

First, the purpose of this study was to understand how flexible and adaptive perception-action couplings, via the QE, may underpin saving actions in skilled football goalkeepers during a representative dyadic task. Second, we attempted to provide an analysis of the QE strategies of individual participants to analyze inter- and intra- individual variability. The rationale for this analysis was to better understand how adaptive variability may have been used by skilled goalkeepers during representative task conditions.

In line with previous work (for example Chia et al., 2017), we found that the typical use of mean values for the QE was not necessarily a prominent characteristic of successful performance within this group of skilled goalkeepers. These findings fall in line with recent work by Ramsey et al. (2020), illustrating how goalkeepers during a penalty kick utilized a range of different QE durations during successful trials. In our work, the QE duration did not appear to be an invariant feature of gaze at the group mean or individual level (Table 1). Marginal differences between saves and goals (Goalkeeper 1) and larger differences between saves and goals (Goalkeeper 4) equally had no significant performance effect.

The timing of the QE, however, has been recognized as a more consistent feature when identifying successful performance (e.g., Vine et al., 2017). During saving actions, the goalkeepers typically drew on a later QE, compared to trials ending in goals. In our findings the QE fixation tended to emerge at the latter stage of the shooter’s preparation to strike the ball and was maintained throughout the shooter’s movements and during ball flight. This strategy appears typical when intercepting fast approaching objects, where individuals have been seen to engage in later visual tracking onsets (e.g., see Land and McLeod, 2000; Croft et al., 2010). This is indicative of skilled individuals prospectively controlling their actions during interceptive actions. For example, Oudejans et al. (2002) found that the availability of later visual information underpins successful performance, allowing individuals to continuously control their actions by maintaining direct contact with the available visual information throughout the action.

### Skilled Goalkeeping May Be Predicated on Actualizing Affordances

Typically, the QE has been founded upon assumptions from a computational paradigm. Indeed, Vickers (1996) hypothesized that a sustained QE duration “plays a key role in the optimal organization of the neural structures underlying this skill” (p. 352). A sustained fixation during the preparation phase supports the construction of an internal representation that programs the initial parameters of the motor-action. As the motor-action is executed Vickers (1996, p. 351; citing Schmidt, 1988; p. 22) concludes that “although the program was organized and most of the work of controlling the skill accomplished, sensory information and in particular vision… can modify the central command structure as the movement is unfolding.” Because the parameters of the movement have been programmed, visual attention is not necessary during the execution phase for successful performance (Williams et al., 2002). However, more recent work and further corroborated by our findings here, have provided evidence that skilled performers remain in constant contact with the visual environment as they modulate their actions throughout the full execution of the task. For example, Vine et al. (2013) when examining a golf task, found that when a short putt was missed it was due to the QE attenuating early. During the final missed putt, there was a shortening of the final QE duration, showing a breakdown in online-control processes. In addition, Vine et al. (2017) occluded visual information during a golf putting task. Whilst no effect was found for occluding early visual information, the occlusion of later visual information led to detrimental performance outcomes. An online control mechanism highlights the significance of a more constant perception-action cycle where performance is controlled online through perceiving relevant visual information and is an important factor in considering how skilled performers control their movements.

Whilst the QE is currently grounded firmly within a computational paradigm, the phenomenon it describes (stillness of the eyes during execution of a goal directed movement) may benefit from a framework that more comprehensively addresses how one constantly modulates their behavior throughout the course of a skilled action. As proposed first by Davids and Araújo (2016) and further acknowledged by Renshaw et al. (2019), the QE in its current form does not currently provide a clear account explaining how one comes to attend to a certain perceptual variable at any given time.

In answer to this call, an *Ecological Dynamics* framework Handford et al. (1997) can provide an exciting new theoretical explanation of the QE phenomenon in skilled performance. A central tenet of Ecological Dynamics, founded upon the work of Gibson (1966), Gibson (1979) is the role of optical information within the visual field, and the specifying nature of perceptual invariants that invite behavior. Gibson termed these invitations *affordances*, a term which captures how behavior is controlled through the functional and reciprocal relationship between an individual and their environment. The use of affordances is actualized in our analysis, revealing how each goalkeeper modulated their actions around the constraints imposed on them by using different information sources. The goalkeepers used two different points of interest to anchor their QE fixation; drawing on the ball or the VP. As illustrated by our simple linear regression model, the specific location the QE fixation was drawn to was likely specified by the timing of the QE fixation. For example, an earlier QE fixation more frequently led to the QE stabilizing at the VP compared to a later fixation attending to the ball.

A key concern in the ontology of affordances is how an individual’s action capabilities (effectivities) constrain the perceptual-motor workspace (Hristovski et al., 2006; Pacheco and Newell, 2018). Previous work has illustrated how individual constraints cause differing relations with information for affordances. Van der Kamp et al. (2018) illustrated how goalkeepers scale their maximum action capabilities to saving actions. Central to this view is the idea that individuals move in order to maintain their interaction with an affordance (Michaels and Oudejans, 1992).

In line with this suggestion, we are able to propose some speculative associations here. In our analysis goalkeeper 1 and 2 utilized fixations at the VP more often, and Goalkeeper 3 and 4 attended to the ball more. It is apparent that faster goalkeepers in our study used the ball more frequently as their speed of movement (evidenced in the Rt and Mt relative% movement phases) allowed them to wait until later to make use of information surrounding ball velocity and trajectory in order to perceive stop-ability. The GPrep phases were longer for Goalkeeper 3 and 4, than for 1 and 2 (Figure 5). Similarly, the Rt of Goalkeepers 3 and 4 were shorter than 1 and 2 (Figure 6). Goalkeepers who typically spent longer in the GPrep stage, had shorter Rt’s, and exploited affordances invited by the moving ball. Information provided by the ball occurs later in the trial and would specify the unfolding trajectory opposed to the information variables provided from the VP. Analyzing the individual goalkeeper’s movement profiles reveals broad differences from the reported mean, demonstrating that the unique individual perceptual-motor profiles are more revealing of how skilled goalkeepers interact with their environments. For example, Goalkeeper 2 varied broadly, where in trial 3 the goalkeeper spent 35.91% of the total movement time waiting in the GPrep phase, however, in trial 9 the GPrep phase lasted as long as 49.54%. Contrastingly, the mean value for Goalkeeper 2 for GPrep is 43.43%, demonstrating wide variability from the mean. This finding, and the intra-individual variability present demonstrates how goalkeepers interact differently with their environments. Specifically, the expert goalkeepers within our sample modulated their movements based on the demands of the task, by waiting longer (GPrep) before moving at greater speed to intercept the ball (Mt) may illustrate how goalkeepers are regulated by the availability of visual information in respect to their own effectivities.

**FIGURE 5:** Each individual goalkeeper’s relative (%) time spent in GPrep movement phase and distribution of trial-by-trial inter-individual data.

**FIGURE 6:** Each individual goalkeeper’s relative (%) time spent in Rt movement phase and distribution of trial-by-trial inter-individual data.

This finding may provide significant considerations for the future of QE analysis. As illustrated by Button et al. (2002), subject by subject analysis can reveal how different control strategies are used during interceptive tasks. In their research, Button et al. (2006) found that certain participants moved earlier, therefore changing the relative timing of the grasp phase, indicating different solution strategies occurring under the manipulation of task constraints. Similarly, Al-Abood et al. (2001), in an under-arm dart aiming task, required participants to learn the skill through either modeling or verbal direction. Analyzing the individual profiles of each participant illustrated how, despite generalized mean findings between intervention groups, some participants whose movement was closer to the relative motions of the model scored better, whereas some participants seemingly scored lower. The variability evident within our analysis may be indicative of the use of functional adaptive variability within their visual search strategies, as opposed to generalized behaviors that treat a group of skilled performers as a single homogenous group.

### Skilled Goalkeeping as the Mastering of a Functional Individual-Environment Fit

In our case study, we have been able to demonstrate incidents of inter-individual variability of the QE within skilled football goalkeepers. To capture the intra-individual variability, and thereby incidents of adaptive variability, Figure 3 illustrated each individual trial respective of fixations at the VP (Figure 3A) and ball (Figure 3B). Similar to the reporting of group mean data, the presentation of individual mean data may also fail to capture how participants form skilled perception-action couplings. Specifically, each individual goalkeeper reported large relative standard deviations (Table 1) from the mean for both onset and offset, illustrating how the timing of the QE fixation may differ in response to emerging constraints upon the task. Each trial can be examined as a separate event due to the emergence and decay of performance constraints occurring within the goalkeeper-kicker dyadic system, consequently leading to unique task solutions (Latash and Anson, 1996). Each individual forms their own signature perception-action coupling through a flexible and adaptable relationship with the dynamics of the task. As noted by Savelsbergh et al. (2004), an individual’s practice history or specifically, his or her exposure to differing constraints during perceptual development may form a variety of different perception-action couplings between individuals of a similar skill level. Through one of Gibson (1979) central concepts to perceptual learning, the education of attention, individuals are able to attune to perceptual invariants in the visual field allowing them to first learn, and then exploit the action-specifying, from non-specifying sources of information (Dicks et al., 2009; van der Kamp and Renshaw, 2015). Our analysis reveals that the timing of the QE fixation varies from the mean in response to the interaction of different constraints; be it task, environment or individual (Newell, 1986; Rienhoff et al., 2016). This in turn affords skilled performers the opportunity to exploit an array of action-specifying variables, forming a functional individual-environment fit. As noted by Dicks et al. (2017) and further substantiated by our findings, it is likely that the interactions between the goalkeeper, their opponent and the environment may mean an information source in one trial, may not emerge or may not be a successful determinant in the next trial. Evidence of this emerges within a trial-by-trial analysis, whereby the goalkeepers flexibly adapted the QE strategy deployed, as well as the specific information variable the QE fixation attended to. With each individual expert performer having his or her own unique information QE profile (Figure 4), the data from the current analysis suggests the need pursue individual analysis of QE strategies of single subjects within their natural performance context in order to more appropriately understand how performers uniquely differentiate themselves.

## Conclusion and Future Implications

### Case-Study Considerations and Future Directions

Before proceeding, we must highlight the cautionary tales of our approach. Whilst we have provided an insight into the natural perceptual behaviors of elite football goalkeepers, we have been constrained by the organizational demands that occur within elite sport environments (Drust and Green, 2013). Access to participants, particularly goalkeepers, are already a smaller subset of the already small elite football population. As the research occurred at the regular training time and at the respective training environments of the goalkeepers, significant time constraints imposed on the availability to collect data. Whilst all clubs were fully supportive of our endeavor, organizational demands often took priority. In light of this, we acknowledge the limitations in the sample and trial sizes. We do not seek to widely generalize these findings; however, we believe that our case study has allowed us to commit to further exploring the case of functional variability present in goalkeepers QE behaviors.

An analysis of individual performers on a single subject basis has emerged as an alternate frame of analysis to capture how variability is a functional component of skilled behavior. Using individual coordination profiling, researchers have been able to illustrate the specific coordination patterns over the course of a movement (Button et al., 2006). For example, Button and Davids (1999) illustrated inter-trial and inter-individual variability in one handed catching where individual kinematic analysis revealed systematic condition effects. When auditory information was removed, participants altered the opening of the hand, the velocity of the wrist or the location of ball-hand contact. However, no effect was illustrated at the group level.

Adopting an individualized profiling approach, it has been possible to capture variability for the QE during skilled performance. Where typical analysis of the QE has tended to assume the group mean data is reflective of all trials, and therefore successful or unsuccessful performance, variability around the mean may in fact show how the QE is a flexible and adaptive perceptual tool.

### Summary

In conclusion, we sought to understand how the QE may function in skilled football goalkeepers via incidents of adaptive variability, evidenced by successful performance that falls away from the mean. We have firstly illustrated how the timing of the QE may provide the athlete with a continuous perception and action cycle as they prospectively control the execution of a goal-directed movement. Secondly, we illustrate how goalkeepers form skilled perception-action couplings, via the QE, opposed to optimal gaze patterning. Specifically, data falling either side of the mean may illustrate how QE patterning emerges through the performer-environment relationship.

Future work in this domain should continue to pursue individual analyses and single subject designs in order to further study inter- and intra- individual variability in participants ranging in skill level, across tasks ranging in complexity. With a clearer understanding of the role variability plays in QE behaviors, practitioners and researchers alike can continue to pursue the merits of QE training programs in upskilling lower skilled athletes.

## Data Availability Statement

The raw data supporting the conclusions of this article will be made available by the authors, without undue reservation.

## Ethics Statement

The studies involving human participants were reviewed and approved by the Oxford Brookes University—DREC Reference 0417-42. The patients/participants provided their written informed consent to participate in this study.

## Author Contributions

BF: conceptualization, methodology, investigation, and writing. WR: conceptualization, supervision, writing—original draft. JJ: supervision and formal analysis. JS: formal analysis, writing—review and editing. KD: conceptualization, writing—original draft, review and editing. All authors contributed to the article and approved the submitted version.

## Conflict of Interest

The authors declare that the research was conducted in the absence of any commercial or financial relationships that could be construed as a potential conflict of interest.

## Publisher’s Note

All claims expressed in this article are solely those of the authors and do not necessarily represent those of their affiliated organizations, or those of the publisher, the editors and the reviewers. Any product that may be evaluated in this article, or claim that may be made by its manufacturer, is not guaranteed or endorsed by the publisher.
